# Construction of a Computer-Aided Analysis System for Orthopedic Diseases Based on High-Frequency Ultrasound Images

This article has been retracted.

**DOI:** 10.1155/2022/8754693

**Published:** 2022-01-05

**Authors:** Feifei Xiu, Guishan Rong, Tao Zhang

**Affiliations:** ^1^Ultrasound Department, The Fourth People's Hospital of Langfang, Langfang, Hebei, China; ^2^Second Department of Orthopedics, The Fourth People's Hospital of Langfang, Langfang, Hebei, China

## Abstract

The area of medical diagnosis has been transformed by computer-aided diagnosis (CAD). With the advancement of technology and the widespread availability of medical data, CAD has gotten a lot of attention, and numerous methods for predicting different pathological diseases have been created. Ultrasound (US) is the safest clinical imaging method; therefore, it is widely utilized in medical and healthcare settings with computer-aided systems. However, owing to patient movement and equipment constraints, certain artefacts make identification of these US pictures challenging. To enhance the quality of pictures for classification and segmentation, certain preprocessing techniques are required. Hence, we proposed a three-stage image segmentation method using U-Net and Iterative Random Forest Classifier (IRFC) to detect orthopedic diseases in ultrasound images efficiently. Initially, the input dataset is preprocessed using Enhanced Wiener Filter for image denoising and image enhancement. Then, the proposed segmentation method is applied. Feature extraction is performed by transform-based analysis. Finally, obtained features are reduced to optimal subset using Principal Component Analysis (PCA). The classification is done using the proposed Iterative Random Forest Classifier. The proposed method is compared with the conventional performance measures like accuracy, specificity, sensitivity, and dice score. The proposed method is proved to be efficient for detecting orthopedic diseases in ultrasound images than the conventional methods.

## 1. Introduction

The most frequent bone condition is osteoporosis. It is a fundamental bone sickness portrayed by diminished natural and inorganic parts of bone tissue per unit volume, which prompts expanded bone construction delicacy and weakness to foundational bone illness described by cracking. The problem of osteoporosis has gotten more prevalent as the population of the elderly continues to expand. This is not only a health issue but also a societal issue that must be addressed. Invasive and noninvasive examinations are the most common clinically helpful procedures for diagnosing osteoporosis in recent years. Noninvasive examinations include biochemical examinations, medical imaging, and bone density assessment. Invasive examinations are primarily based on histomorphometry. For osteoporosis, there are a variety of imaging diagnostic modalities available, such as QCT (quantitative computed tomography) [1], UTE (ultrashort echo) [2], DWI (diffusion-weighted imaging) [3], DXA (dual-energy X-ray absorptiometry) [4], and QUS (quantitative ultrasound) [5]. For the diagnosis of osteoporosis by BMD (bone mineral density), DXA is the “gold standard.” At this point, it has become a generally accepted diagnostic tool.

DXA works on the same X-ray principle as before. This technique differs because it uses high- and low-energy rays to determine tissue density and generate distinct attenuation distribution curves. The scientists need to enter the acquired bend into the PC for present handling to get the bone mass per unit region, to be specific, BMD (bone mineral density). The most common DXA measuring positions are the thoracic vertebrae and the highest reaches of the femur. Even though DXA is this double intersecting image, it cannot distinguish among bones of cortical and cancellous nor can it deal with artifacts caused by interlacing soft tissue in the spinal column, both calcification such as abdominal and aortic and so on, and a variety of factors influence BMD measurement accuracy. Quantitative computed tomography (QCT) is a much more sophisticated sensor module that can assess the cortical bone mineral density and the cancellous bone mineral density and volume BMD. At the moment, DXA offers clear benefits in terms of evaluating BMD, which is an essential criterion for determining osteoporosis and injury risks. The results produced by measuring BMD by QCT are very comparable with DXA, according to numerous studies. The advantage is that there is no overlapped impact, but the patient receives a higher radiation dosage and a reasonably high examination cost. Therefore, the clinical use is limited. Ultrasound (US) systems send and receive sound pulses through the body of the patient. These systems are frequently used because of their significant benefits, including the lack of radiation and low cost. Compared to other methods such as magnetic resonance imaging or computed tomography, on the other hand, they produce low-quality images. The low quality is primarily associated with multireflections of the signals, which results in so-called speckle noise, which lowers brightness, degrades features, and reduces overall image resolution. To overcome this problem, ultrasound (US) is the most straightforward clinical imaging tool. Hence, it is widely employed in healthcare and medical settings that use computer-assisted systems shown in Figure 1.

We suggested a three-stage segmentation approach for orthopedic disease US pictures in this study, in which abnormalities are recognized first, then segmented. Both identification and segmentation networks are built using the U-Net architecture, which has been shown to train quickly and with few images. According to our hypothesis, it will improve the efficiency of the segmentation network by decreasing the candidate region.

The proposed methodology contribution is as follows:

- To enhance the frequency image and noise-free image, Enhanced Wiener Filter is used in the preprocessing step
- Three-stage image segmentation was introduced using U-Net to detect orthopedic diseases in ultrasound images efficiently
- The transformation-based analyzer technique is used to enhance feature extraction
- To reduce the optimal subset, the Principal Component Analysis (PCA) Algorithm was used
- To enhance the classification stage very efficiently, the Iterative Random Forest Classifier Algorithm was used

The remaining section can be organized in the following manner: Section 1 is the introduction of computer-aided diagnosis system for orthopedic diseases.  Section 2 describes the related work.  Section 3 includes a detailed illustration of the actual system design. In Section 4, the procedures were validated with orthopedic US datasets and presented the findings. In Section 5, finally, we concluded the study.

## 2. Related Works

The U-NET network is used in this paper to offer an improved osteoporosis detection algorithm. To begin, the original image's bone is obvious with second-hand to create dataset. Normalizing each layer's input, the hidden layer distributions of each layer may be assumed to be stable, allowing the goal of rapid training to be attained [6, 7]. Computer-assisted diagnosis methods in orthopedic surgery have shown promise in mechanically identifying and detecting fractures. Using a mix of sliding window techniques and support vector machines, this work presents a system that automatically recognizes and identifies the diaphyseal femur fractured component in X-ray pictures. Orthopedic surgery and therapy are concerned with the human muscular system. Degenerative diseases, injuries, sports injuries, malignancies, and congenital problems are all part of it. Orthopedic surgeons are constantly eager to obtain an X-ray image of a patient's injured body parts to provide a more accurate diagnosis. Electronic radiation is sent through the human body during X-ray imaging to get bone images. A doctor manually checks an X-ray image after it has been retrieved. [8] used an X-ray image to detect several orthopedic and radiology-based mussel diseases in this study. Average, middle, and Wiener filters are employed to remove noise in the preprocessing stage; edge detection recognition is suggested for image capture. Radial basic function (RBFNN) deep learning optimization is devised for disorder classification [9]. The use of a T2-weighted sagittal MR scan to diagnose degenerated discs is presented as an automatic diagnostic system. To segment the lumbar IVD from either a midsagittal MR picture, a completely automated Expectation-Maximization- (EM-) based novel IVD segmentation is suggested. Then, from segmented IVDs, Gabor features, a blend of basic brightness and constant moments, are recovered [10]. The support vector machine (SVM) classification is used to categorize IVDs as degenerate or non-degenerate. For 93 clinical sagittal MR pictures of 93 cases, the suggested system was trained, tested, and reviewed [11]. The trade-off between volume and veracity in X-ray image-based bone fracture categorization is investigated in this study. The effects of using Principal Component Analysis as a compression tool to reduce dimensionality on X-ray picture categorization are investigated. The biggest issue with X-ray pictures is that they might be blurry, out of focus, too bright, or too loud, making scrutiny complicated [12]. To aid ultrasound operations in detecting rotator cuff diseases and increase the feasibility of ultrasound testing, a computer-aided diagnostic (CAD) process was built. There were 43 cases of irritation, 30 cases of intra-articular tendinitis, and 26 tears among the patients collected. The disease area and feature descriptors from the whole lesions were retrieved and merged in multiple logistic regression classifiers for lesion categorization for each case [13]. To improve the diagnosis, a computer-aided diagnosis (CAD) system was created to aid in the effective segmentation and three-dimensional restoration of the lateral epicondyle tendon. The created CAD system would offer data on the input dataset, segmentation findings, and data methods of the damaged anterior cruciate ligaments [14]. For multiple training procedures, two modeling strategies were used. The training was meant to be feasible even with a minimal amount of information, based on the outcomes of the initial transformation. The model's efficiency by using the horizontal flip, rotations, breadth, and altitude shift algorithms was improved [15]. A computer-aided diagnosis (CAD) method for identifying multiclass kidney problems from ultrasound pictures is proposed in this research. The CAD system extracts features using a pretrained ResNet-101 model and classifies them using a support vector machine (SVM) classifier. Ultrasound images are frequently influenced by speckle noise, which reduces data quality and CAD system efficiency [16]. To identify bone fractures in human fingers via image analysis, we developed and tested an approach. A major drawback of X-ray pictures is that they may distort them and be out of focus, too noisy, and bright, all of which make inspection harder since they obscure details [17]. For the current method, complex structural structures are represented using implicit modeling tools derived from the reconstruction of anatomic CT images. [18] suggested that students take a problem-based training course that included the NESTOR program. The students were given written exams during the course that they had to complete before and after the course. They also had to complete an objective structured clinical examination (OSCE) and a questionnaire for their assessment after finishing the course [19]. Ultrasound bone identification and worldwide CT registrations have both been automated completely by our techniques. An in vivo spine feature representation in the bone identification method was used, which was then extensively tested on both datasets which are ex vivo and in vivo. [20] used skeletal patchwork from radiography of a spinal model to train a DNN. It was possible to determine the Cobb angle of the spinal curve by using the projected vertebral slopes from the deep neural network. In vivo radiography from 65 patients and model radiography from 40 patients examined each. The radiography in question was measured by hand by an accomplished surgeon. To evaluate the above radiography, two examiners utilized both the suggested and subjective measuring techniques. [21] present nonlocal median filtering. The CAOD method minimizes distortion and divides DXA pictures, allowing it to identify areas of interest better. A pixel is classified as being either bone or soft material using a pixel labeling random forest. Afterward, based image contours are used to identify areas of interest and compute BMD using soft tissue pixels [22]. Picture features may be retrieved using a Harris corner-based detection method that identifies the presence of edges, fractures, and corners. This technique can extract image features. Osmania Health Center in Hyderabad has provided us with 300 different X-ray pictures [23]. Medical picture segmentation is a good application for the suggested techniques because of the benefits that may be seen. In terms of picture similarity, the Haar wavelet had the best results. The wavelet transform method can deconstruct X-ray pictures using the finely detailed horizontal, vertical, and diagonal parts [24]. We provide 2 novel different crack detection methods in this article. First, we use Faster Area with Convolutional Neutral Network (Faster R-CNN) to identify 20 distinct kinds of bone areas in X-ray images and then CrackNet to determine whether or not each bone region is broken [25]. As a key piece of intelligent equipment to aid in developing precise and minimally invasive orthopedics surgery, orthopedic surgical robots have drawn considerable attention from researchers worldwide. This chapter provides an overview of orthopedic surgical robot development as well as common orthopedics robot products.

## 3. Proposed Work

The research framework for a computer-aided diagnosis system for orthopedic illnesses recognized effectively or not in ultrasound pictures has been implemented in this section.  Figure 2 shows a schematic illustration of the planned flow.

- MURA Orthopedic dataset

The labeled exams submitted to the network made up the training MURA dataset. The testing set was chosen randomly from the original dataset and was never utilized during training or validation. 76% of fractures are detected. Iterative Random Forest Classifier (IRFC) classified and validated the test dataset individually and separately, using the same framework as the training dataset.

### 3.1. Preprocessing

#### 3.1.1. Enhanced Wiener Filter

The Enhanced Wiener Filter is a Wiener filter that is proposed. By presenting the modification of the filter intensity to the local properties of the image, the method solves one of the Wiener filter's fundamental limitations. The MRF Markov Random Field theory was adopted to model the noise-free image and then optimize the filtration intensity achieves this characteristic. The technique incorporates computational time efficiency, excellent denoising results, and low supervision requirements. Take a look at the acquisition model below:

(1) $$\begin{array}{c} a\left(z,s\right)=x\left(z,s\right)\;n\left(z,s\right), \end{array}$$

where *a*(*z*, *s*) is the data acquired, *x*(*z*, *s*) is the noise-free signal, and *n*(*z*, *s*) is the speckle noise.

The multiplicative structure is transformed into additive using a logarithmic conversion, yielding

(2) $$\begin{array}{c} r^{\prime }\left(z,s\right)=\log\left[a\left(z,s\right)\right]=\log\left[x\left(z,s\right)\right]+\log\left[n\left(z,s\right)\right],\\ r^{\prime }\left(z,s\right)=x^{\prime }\left(z,s\right)+n^{\prime }\left(z,s\right). \end{array}$$

### 3.2. Image Segmentation in Three Stages Using U-Net and Test Time Augmentation (TTA)

#### 3.2.1. First Stage of U-Net Segmentation

Here, we proposed U-Net architecture in segmentation of US images. The network's contraction section comprises three convolutional layer blocks with ReLU activation, accompanied by a max-pooling procedure shown in Figure 3. The network is symmetric, and the expansion phase includes blocks of two convolutional layers followed by an upsampling process. By concatenating the learned characteristics from the contraction phase to the expansion part, some skip connections transport information from the contractions part to the growth part. There are 64 filters in the first three convolutional layers. After each max-pooling process, the number of filters doubles by three in the contraction section. After each upsampling operation, the number of filters drops by a factor of three in the expansion section.

#### 3.2.2. Second Stage and Third Stage of U-Net Segmentation

In this research, we proposed that the same network (U-Net) be used for both the ROI identification and segmentation stages for orthopedic US pictures. Our study suggested a framework's overall design consists of three U-Nets, the first responsible for detecting where the lesion exists, the second for segmenting the detected region, and the third for segmenting the region portion normality or abnormality. We created a new ground truth based on the previous surrounding truth to train the first network instead of the real lesions form; we used the surrounding area. The network was then trained in the same manner as the one-stage technique, using a five-fold bridge with the same termination conditions, pretrained weights, and model of society ratio. Then, at that point, the yield of the primary organization was considered the contribution for the subsequent organization, and the yield of the second organization was considered the contribution for the third organization. The discovered regions' enclosing area was cropped, then sent to a second network to be split, and the normalcy of region component was detected. If the first network recognized more than one distinct region in a single image during training and testing, all detected regions were treated as input to the second network. The third network detected normality and abnormality (Figure 4).

#### 3.2.3. Test Time Augmentation (TTA)

The segmentation of the second and third stages of network performance is dependent on how successfully the first network detected the lesion location. The second network will be able to segment the image precisely if the first network recognizes the square correctly and the third network detects the abnormality of the lesion. On the other hand, the second network will fail if the detection step fails and the lesion is missed, or only a portion of the lesion is detected. As a result, an approach for determining if the detection stage functions correctly and whether the detection results are valid is required. We recommended utilizing the test-time augmentation technique in two distinct ways to examine this. First, we alter the test data to supplement it. We can expect the identified region to move in the same direction as the image is shifted for a few pixels if the detection is done correctly. If the detection is unstable, however, the detected region is likely to vary in an unforeseen way. As a result, we moved the picture for ten various values (15, 20, 25, 30,…, -30, -25, -20, -15) of pixels and looked at how the identified region altered as a result.

At the test time, we applied the dropout approach as the second method. In deep learning, dropout has been proven to represent model parameters. The network is supposed to produce somewhat different results each time it is run by using dropout at the test time. The result is regarded as questionable when there is variability between multiple ranges for the same input. If the model produces a high-uncertainty output, it may be worthwhile to validate it further. We computed the production of the detection network by each picture in the testing sample 10 times, maintaining the automatic dependent active at the test time.

In the same way, we computed the output of the shifting operation. The detecting network is regarded as valid when the uncertainty between different runs is low. The uncertainty between different runs was measured using the Dice score. Obtain the Dice score by comparing the network output when the dropout layer was eliminated to the network output when the dropout layer was active. The performance of the first network is regarded as faulty when both techniques proclaim the outcome to be an invalid result.

### 3.3. Feature Extraction

The process of obtaining quantitative information from the image, like color properties, structure, size, or contrast, is known as feature extraction. The DWT (Discrete Wavelet Transform) was used to extract wavelet coefficients, and GLCM (Gray Level Cooccurrence Matrix) was used to extract statistical features. Using multiple scales, the wavelet was utilized to evaluate distinct frequencies of an image. We are using the DWT (Discrete Wavelet Transform), which is a valuable technique for extracting features and used it to derive wavelet coefficients from orthopedic imaging features are listed as follows:

#### 3.3.1. Contrast

Above the image, the equation is used to calculate the pixel intensities and their neighbors.

(3) $$\begin{array}{c} C=\overset{x-1}{\underset{a=0}{\sum }}\overset{y-1}{\underset{b=0}{\sum }}{\left(a-b\right)}^{2}g\left(x,y\right). \end{array}$$

#### 3.3.2. Energy

The quantity of repeating pixel pairings is defined by energy. It is the mathematical expression for the measurement of affinity in an image.

(4) $$\begin{array}{c} E=\sqrt{\overset{j-1}{\underset{m=0}{\sum }}\overset{k-1}{\underset{n=0}{\sum }}g^{2}\left(m,n\right)}. \end{array}$$

#### 3.3.3. Correlation

The measuring of pixel-to-pixel spatial feature relationships is as follows:

(5) $$\begin{array}{c} C_{r}=\frac{\sum_{m=0}^{j-1}\sum_{n=0}^{k-1}\left(m,n\right)g\left(m,n\right)-P_{m}P_{n}}{\sigma_{m}\sigma_{n}}. \end{array}$$

#### 3.3.4. Homogeneity

In an image, it measures the local uniformity. Also, it is called the inverse difference instant, and it has a simple or complex value range to differentiate involving surfaces.

(6) $$\begin{array}{c} H_{o}=\overset{j-1}{\underset{m=0}{\sum }}\overset{k-1}{\underset{n=o}{\sum }}\frac{1}{1+{\left(m-n\right)}^{2}}g\left(m,n\right). \end{array}$$

#### 3.3.5. Entropy

It estimates the orthopedic image's designated interference. It is written as

(7) $$\begin{array}{c} E_{NT}=-\overset{j-1}{\underset{m=0}{\sum }}\overset{k-1}{\underset{n=0}{\sum }}g\left(m,n\right)\log_{2}\;g\left(m,n\right). \end{array}$$

The following feature assessment parameters must be obtained for better interpretation of Orthopedic US images.

#### 3.3.6. Peak Signal-To-Noise ratio

It is a metric for evaluating the characteristics of a reconstructed image derived from an input image.

(8) $$\begin{array}{c} \text{PSNR}=20\;\log_{10}\frac{2^{n}-1}{\text{MSE}}. \end{array}$$

#### 3.3.7. Mean Square Error

Signal or picture fidelity is measured. We used it to compare two photos by assigning numerical or similarity ratings to them.

(9) $$\begin{array}{c} \text{MSE}=\frac{1}{R\times S}\sum \sum {\left(g\left(x,y\right)-g^{2}\left(x,y\right)\right)}^{2}. \end{array}$$

These statistical variables were supplied into the Iterative Random Forest Classifier (IRFC) as an input for testing and training the classifier's effectiveness in separating abnormal and normal orthopedic pictures.

### 3.4. Feature Selection

This section outlines the PCA-based feature selection technique that is recommended. The goal of feature selection, since we all understand, is to limit the number of measurements. We begin with selecting features PCA-based. We understand that the feature selection outcome of an arbitrary sample vector *b*, with regard to *z*, is if *x* is an eigenvalue of the covariance of PCA.

(10) $$\begin{array}{c} X=b^{T}z=\overset{N}{\underset{j=1}{\sum }}b_{j}z_{j}, \end{array}$$

where *z* is the [*z*_1_, ⋯,*z*_*n*_]^T^, *b* is [*b*_1_, ⋯,*b*_*n*_]^T^, and *n* is the dimensional sample vector.

The absolute value of *z*_*j*_ (*j* = 1, 2, ⋯, *n*) can be used to statistically analyze the impact of the *j*th feature element of data on the outcome of the extracting feature. We can quickly diagnose the absolute smaller value of *z*_*j*_ and *i*th feature components of less contribution. However, eliminating *b*_*k*_*z*_*k*_ from ∑_*j*=1_^*n*^*b*_*k*_*z*_*k*_ will almost not influence the feature extraction outcome if the exact amount of *z*_*k*_ is small enough.

We can assume that if a feature component is not crucial for feature extraction, it is likewise not relevant in the original space. As just a consequence, if the exact amount of *z*_*k*_ is small enough, the *k*th feature component of samples might be considered unimportant and removed. We also recognize that there are always many eigenvectors. Thus, we recommend considering multiple eigenvectors when assessing the relevance of a single feature component.

### 3.5. Iterative Random Forest Classifier (IRFC)

Nonlinear classifiers made out of many decision trees are known as random forest classifiers. The average prediction of the forest's trees is the forest's production. Each tree is trained on a collection of characteristics and data to guarantee that the trees are suitably distinct. Each tree is made up of a sequence of nodes, each of which can either branch into two child nodes or be a leaf node using a splitting rule. A splitting authority is derived for each yet-to-be-split node that best differentiates the favorable and unfavorable samples that arrive at that node while learning the forest. The fresh sample is sent through every tree according to splitting criteria at test time, eventually ending in a leaf node. The fraction of successful training images at that leaf node determines the output value of sampling from a tree. Random forest classifiers operate well with a subset of features. They have a fundamental feature selection property that allows them to choose the optimal feature during training for dividing each node. This qualifies them for patch-based learning, which is what we suggest for US classification. All pixels in a three *n* window surrounding a US pixel are considered feature candidates in this study. For prediction tasks, the IRF is a predicting and interpretable approach. While the IRF is more accurate than other traditional prediction techniques, it has a computational cost with random forests. In this paper, the iterative random forest algorithm is used to detect tumor types in orthopedic dieses.

## 4. Performance Analysis

### 4.1. Accuracy

Accuracy is a statistic that may be used to analyze the outcomes of machine learning techniques. Because their working mechanisms differ, the accuracy of the different algorithms in this study varies slightly. The Accuracy AUC is determined by the number of adequately identified targets and is calculated using the following formula:

(11) $$\begin{array}{c} \text{AUC}=\frac{tp+tn}{tp+tn+fp+fn}. \end{array}$$

The comparative analysis of accuracy, sensitivity, and specificity is shown in Table 1.

When compared to other methodologies, our proposed method received the highest accuracy score.  Figure 5 depicts the accuracy of the four approaches. In this graph, the *X*-axis contains data and *Y*-axis includes the accuracy range. Because we use ultrasound images to identify orthopedic problems, our suggested technique provides better outcomes than previous methods.  Figure 6 depicts knee detection.

### 4.2. Sensitivity

Sensitivity is defined as the percentage of positives that are appropriate implementation as positives.  Figure 7 shows that the sensitivity.

(12) $$\begin{array}{c} \text{Sen}=\frac{tp}{tp+fn}. \end{array}$$

### 4.3. Specificity

Specificity refers to the percentage of negative specimens that are correctly identified.  Figure 8 shows that the specificity result.

(13) $$\begin{array}{c} \text{Spe}=\frac{tn}{tn+fp}. \end{array}$$

### 4.4. Dice Score

In this proposed system, the three-stage U-Net algorithm detects the orthopedic dieses from ultrasound images.  Figure 9 displays some photos where the lesions were not discovered using the one-stage method. Next, we divided the photos into three groups based on the segmentation findings of the one-stage method's weak and robust performance. We defined poor segmentation as having a Dice score of less than 72%, including images with undiscovered lesions (Dice score = 0). The average Dice score was 35.3 percent, while 32 photos had a Dice score below 72%. The average Dice score climbed to 49.9% when used the two-stage strategy, and 16 of the 32 photos got a Dice score of more than 72%. Only three of the 32 images had inferior outcomes when used the two-stage approach. In three stages, the lesion detects the normality or abnormality of keen detection.

We utilized Dice score, which is a metric of overlapping between the segmented region and the surrounding area, to estimate the accuracy of the segmentation outputs of the three algorithms discussed above the definition of the surrounding:

(14) $$\begin{array}{c} \text{DS}=\frac{2\times \text{True Positive}}{2\times \left(\left(\text{True Positive}\right)+\left(\text{False Negative}\right)+\left(\text{False Positive}\right)\right)}. \end{array}$$

Here, True Positive is denoted as the mask, the total number of components properly predicted, False Positive denoted as the number of components that the technique incorrectly identified as the mask, and False Negative denoted as the number of components in the surrounding area mask that the segmentation algorithm fails to detect.

For the various subsets of photos, Table 2 shows the outcomes of one-, two-, and three-stage techniques.  Figure 10 shows the value of the Dice score, in which three-stage part of the Dice improvement can be attributed to the three-stage approach's improved segmentation. Here, the blue bar indicates that nontest time augmentation at the third stage improved the segmentation.

## 5. Conclusion

This paper proposed new approaches for segmentation and classifying orthopedic image detection for deep learning. The suggested U-Net approach and iterative random forest classification model are based on different parameters and iterative by the accuracy measurement. Based on data processing derived by the methods of Wiener filter, preprocess is assessed. When comparing the findings of the different learning models, the suggested IRFC classification accuracy is 95.5%. The proposed classification method is based on random forest techniques. The results show that the proposed approach outperforms existing accuracy, sensitivity specificity, and Dice score.

## Figures and Tables

**Figure 1:** General flow for computer-aided diagnosis.

**Figure 2:** Schematic diagram for the proposed methodology.

**Figure 3:** Architecture for U-Net.

**Figure 4:** Three-stage approach for segmentation detection in orthopedic US image.

**Figure 5:** Comparison of accuracy.

**Figure 6:** Image detection using ultrasound scan.

**Figure 7:** Comparison of sensitivity.

**Figure 8:** Comparison of specificity.

**Figure 9:** Stage-wise lesion detection.

**Figure 10:** Dice score for three-stage approach.

**Algorithm 1:** Iterative Random Forest Algorithm.

**Table 1:** Comparison of classification analysis.

Algorithms	Accuracy	Sensitivity	Specificity
Logistic regression [16]	81	80.8	80
*K*-nearest neighbor [16]	85	84.2	83.2
Random forest [16]	89	88.2	87
Iterative random forest [proposed]	95.5	94	92.3

**Table 2:** Dice score for three-stage approaches.

	All images (non-TTA)	Images with valid detection	Images with invalid detection
One-stage	78.35	83.5	68.8
Two-stage	80.5	87.4	64.2
Three-stage	85.5	89.8	45.1

## Data Availability

The dataset used to support the findings of this study are available from the corresponding author upon request.
